This article has been retracted.

# Influence of Melatonin on Behavioral and Neurological Function of Rats with Focal Cerebral Ischemia-Reperfusion Injury via the JNK/FoxO3a/Bim Pathway

**DOI:** 10.1155/2022/8202975

**Published:** 2022-01-17

**Authors:** Xingwang Chen, Xueyuan Shen, Jianbo Lai, Zhijun Yao, Xian Peng, Long Wu, Yuantong Ou, Huachu Wu, Haofeng Zhu, Yiyu Deng

**Affiliations:** ^1^The Second School of Clinical Medicine, Southern Medical University, Guangzhou, 510515 Guangdong, China; ^2^Department of Critical Care and Emergency, Department of Cardiology, Shenzhen Hospital of Integrated Traditional Chinese and Western Medicine, Shenzhen, 518104 Guangdong, China; ^3^The Second Clinical Medical College, Guangzhou University of Chinese Medicine, Guangzhou, 510515 Guangdong, China; ^4^Department of Critical Care and Emergency, The Second Affiliated Hospital of Guangzhou University of Chinese Medicine, Guangdong Provincial Hospital of Chinese Medicine, Guangzhou, 510515 Guangdong, China; ^5^Furong Community Health Service Center, Shenzhen Hospital of Integrated Traditional Chinese and Western Medicine, Shenzhen, 518104 Guangdong, China; ^6^Department of Critical Care and Emergency, Guangdong Provincial People's Hospital, Guangzhou, 510515 Guangdong, China

## Abstract

**Objective:**

To investigate the influence of melatonin on behavioral and neurological function of rats with focal cerebral ischemia-reperfusion injury via the JNK/FoxO3a/Bim pathway.

**Methods:**

One hundred and twenty healthy male SD rats were randomized into the model group (Model: the middle cerebral artery occlusion (MCAO) model was constructed and received an equal volume of normal saline containing 5% DMSO), sham operation group (Sham: received no treatment except normal feeding), and low, medium, and high dose of melatonin group (L-MT, M-MT, and H-MT intraperitoneally injected 10, 20, and 40 mg/kg melatonin 30 min after IR, respectively), with 24 rats in each group. Following 24 h of reperfusion, the rats in each of the above groups were tested for neurological deficit symptoms and behavioral changes to screen the rats included in the study. HE and TUNEL stainings were performed to observe pathological changes. Levels of oxidative stress-related indexes, inflammatory factor-related indexes, nuclear factor-*κ*B p65 (NF-*κ*B p65), and interferon-*γ* (IFN-*γ*) in the rat brain were measured by ELISA. The JNK/FoxO3a/Bim pathway-related proteins as well as Bcl-2, Caspase-3, and Bax were examined using Western blot.

**Results:**

Detection of behavioral indicators showed that the MACO model was successfully constructed in rats. L-MT, M-MT, and L-MT groups presented reduced malondialdehyde (MDA), reactive oxygen species (ROS), tumor necrosis factor- (TNF-) *α*, interleukin- (IL-) 6, IL-1*β*, IFN-*γ*, NF-*κ*B p65, and apoptosis compared with the Model group (*P* < 0.05), and the improvement degree was better in the M-MT group versus the L-HT group. Bcl-2 protein expression in the brain tissue of L-MT, M-MT, and H-MT groups increased significantly, while Bax, Caspase-3, p-JNK, p-FoxO3a, and Bim protein expression declined markedly, versus the Model group (*P* < 0.05). The changes of indexes were greater in the M-MT group compared with that in the L-MT group. No significant difference was observed in all the above indexes between the M-MT group and the H-MT group (*P* > 0.05).

**Conclusions:**

In the MACO rat model, melatonin can effectively reduce Bax and Caspase-3 levels by modulating the JNK/FoxO3a/Bim pathway, inhibit neuronal apoptosis, and alleviate neurological deficits by reducing the release of proinflammatory mediators, with anti-inflammatory and antioxidant effects. In addition, 20 mg/kg is the optimal melatonin concentration.

## 1. Introduction

Cerebral stroke, also known as stroke [1], is a group of acute cerebrovascular diseases caused by sudden rupture of blood vessels in the brain or inability of blood flow to the brain due to vascular blockage, including hemorrhagic stroke (HS) and ischemic stroke (IS) [2, 3]. The incidence of stroke is increasing year by year worldwide, and the prevalence of IS was higher than that of HS [4]. The mortality/disability rate of patients with acute IS is relatively high, which not only greatly increases the family financial burden and reduces the living ability of the patients but also aggravates the economic and social burden. Therefore, clarifying its pathogenesis and carrying out targeted treatment is of utmost importance.

At present, the treatment of IS is mainly aimed at reperfusion, neuroprotection, and neurological recovery [5]. However, in the reperfusion process of recovering blood flow after cerebral ischemia, it will cause more serious damage to brain tissue, namely ischemia-reperfusion injury (IRI) [6]. Because of the long-term ischemia of brain tissue, local inflammation and reactive oxygen species accelerate to produce when the blood supply returns to normal, which, instead of promoting the recovery of brain function, will aggravate brain injury and capillary dysfunction and lead to secondary brain injury, brain edema, hemorrhagic transformation, necrosis, and free radical injury with infarction growth, resulting in strong neuroinflammatory reaction and even death in severe cases [7, 8]. The formation of focal cerebral ischemia injury is closely associated with neuronal apoptosis [9]. Melatonin (MT) is a tryptophan metabolite released from the pineal gland. As a broad-spectrum antioxidant and an effective free radical scavenger, it plays a neuroprotective role through antioxidant, antiapoptotic, and anti-inflammatory actions, in addition to the function of regulating sleep [10]. Besides, by inhibiting the Rac1/JNK/FoxO3a/Bim pathway, MT can protect cardiomyocytes against oxygen-glucose deprivation and reperfusion [11]. MT has also been correlated with brain damage. Previous literature has reported that the administration of MT after cerebral ischemia can significantly reduce infarct volume [12]. However, the underlying mechanism and pathway of action of MT after cerebral ischemia remain to be further elucidated.

As a member of the mitogen-activated protein kinase family, C-Jun amino terminal kinase (JNK) plays an important role in the regulation of stress, cell differentiation, and apoptosis [13]. In addition, it is shown to be activated in models of neuronal apoptosis under excitotoxicity, nutrient withdrawal, and ischemia inducements [14]. Fork-head transcription factor (FoxO) is the key effector of JNK-mediated tumor suppression [15]. Activation of FoxO regulated by JNK enhances the ability of animals to resist oxidative stress and longevity [16, 17]. It has been reported [18] that fork-head box O3a (FoxO3a) is involved in the myocardial injury process caused by IRI, and the activation of the PI3K/Akt pathway can phosphorylate FoxO3a and transfer it from the nucleus to the cytoplasm to participate in reducing the apoptosis of cardiomyocytes. Meanwhile, the expression of apoptosis regulatory protein Bim, one of FoxO3a's downstream target molecules, is underexpressed. In a neonatal hypoxic ischemia model, Bim, a member of the Bcl-2 family, has been proved to be a critical mediator of neuronal apoptosis [19]. Li et al. [20] found that the JNK/FoxO3a/Bim pathway is involved in rat neuronal apoptosis after hypoxic-ischemic brain injury, and the regulation of FoxO3a by JNK may not depend on Akt. However, the influence of MT regulation of the JNK/FoxO3a/Bim pathway on focal cerebral IRI remains to be clarified. The innovation and significance of our study were to investigate the influence of MT regulation of the JNK/FoxO3a/Bim pathway on focal cerebral IRI, which might obtain some conclusions regarding the mechanism of action of MT on focal cerebral IRI through a new pathway. This study explored the influence of MT on behavioral and neurological functions of rats with focal cerebral IRI via the JNK/FoxO3a/Bim pathway.

## 2. Materials and Methods

### 2.1. Experimental Animals and Groups

Adult healthy male SD rats of SFP grade (body mass: 280-320 g, average weight: 295.72 ± 10.23 g; Animal Laboratory, Guangzhou University of Chinese Medicine) were assigned to the model group (Model), sham operation group (Sham), low dose of melatonin group (L-MT), medium dose of melatonin group (M-MT), and high dose of melatonin group (H-MT) according to the random-number table method, with 24 rats in each group. And the other rats serve as substitutes. The rats were accommodated for two weeks in the environment of room temperature 22-23°C, relative humidity of 45-60%, and 12 : 12 h light-dark cycle. All animal experiments were approved by the relevant ethics committee and were carried out in accordance with the National Institutes of Health guidelines.

### 2.2. Pretreatment of Rats and Establishment of Models

After successful intraperitoneal anesthesia with 1% pentobarbital sodium (40 mg/kg), different operations were performed in each group. An IRI model of middle cerebral artery occlusion (MCAO) was constructed using the modified Longa method [21]. Reperfusion was completed 6 h after ischemia by directly pulling the nylon thread out of the internal carotid artery for about 16 mm, and the anal temperature was kept at 37 ± 0.5°C until 2 h after reperfusion. Criteria for the successful model establishment were as follows: after the rats woke up, the right forelimb curled and flexed after tail lifting and suspension. The rats developed left-sided Horner syndrome and fell to the right side or turned in circles while crawling. Elimination criteria are as follows: rats with subarachnoid hemorrhage, no pathological changes of ischemia, or death at the observation time point were eliminated. In the process of modeling, a total of 11 rats were eliminated, all of which were supplemented by prepared substitutes. Separation of the left common carotid artery as well as the internal and external carotid arteries and suture without nylon thread insertion were performed in the Sham group. MT (Sigma) was dissolved in dimethyl sulfoxide (DMSO, Sigma) and diluted with normal saline to a final 5% DMSO solution. The five groups received the following interventions: L-MT group: intraperitoneally injected with low concentration of MT (10 mg/kg) 30 min after IR; M-MT group: intraperitoneally injected with medium concentration of MT (20 mg/kg) 30 min after IR; H-MT group: intraperitoneally injected with high concentration of MT (40 mg/kg) 30 min after IR; Model group: received an equal volume of normal saline containing 5% DMSO; and Sham group: received no treatment except normal feeding.

### 2.3. Behavioral Tests and Neurological Scores

The behavioral changes of cerebral IRI rats were observed after recovery from anesthesia. The maze (size: 76 cm × 72 cm × 57 cm) was divided into 25 squares. During the test, the rats were placed in the middle of the grid, and the number of squares crawled within 10 min was counted. A consistent lighting intensity and a quiet environment were maintained during each test. The experimental observers used blind test, that is, if the rats showed proper behavior in one evaluation but did not show it later, they were scored according to the previous one. The more grids crawled, the better the neurological function of rats. The method of Longa et al. [21] was used to score the behavior of four groups of rats and record the symptoms of neurological deficit: 0, no behavioral abnormalities; 1 point, the forelimb flexion on the opposite side of the infarct presented a clenched fist; 2 points, muscle strength and lateral thrust were weakened on the contralateral limb of infarction; 3 points, turning to the opposite side or dumping when walking; and 4 points, consciousness disorder, paralysis, or death. Rats with a score of 1-3 were considered successfully modeled and enrolled.

### 2.4. Sampling and Specimen Preparation

Rats in each group were randomized into two groups with 10 rats each. Samples were collected 24 h after reperfusion, some of which were used for HE and TUNEL stainings, and the others for WB and ELISA.

HE staining and TUNEL staining are as follows: 24 h after reperfusion, the rats were successfully anesthetized by routine anesthesia and fixed by paraformaldehyde perfusion. Then, the brain was quickly severed on ice. The cerebral cortex of the ischemic side was fixed in 4% paraformaldehyde for 24 h. After alcohol gradient dehydration, xylene dewaxing, and paraffin embedding, paraffin sections were made with a thickness of about 5 *μ*m. The slices were spread, dehydrated, and baked to make paraffin sections.

Preparation of partial specimens of WB and ELISA is as follows: After 24 h of reperfusion, the brain tissue of rats was quickly and gently removed after routine anesthesia and placed in a Petri dish on ice. Then, a 1-2 mm deep incision was made along the coronal plane of the brain tissue at a distance of about 5 mm along the posterior margin of the cerebral cortex of rats. The tissue near the incision was gently removed with ophthalmic forceps, and the hippocampus was gradually exposed. The complete hippocampus was quickly and gently removed and then placed in a numbered freezing tube, which was quickly placed in the refrigerator at -80°C for cryopreservation.

### 2.5. HE Staining

The paraffin section specimens for HE staining were taken out and placed at indoor temperature for 30 min and then dewaxed in xylene for 5-10 min according to the instructions of HE staining kit (Beyotime Biotech, China). Then, fresh xylene was used for another 5-10 min of dewaxing. After that, they were then dehydrated with anhydrous ethanol, 90% ethanol, 80% ethanol, and 70% ethanol for 5 min, 2 min, 2 min, and 2 min, respectively, and then rinsed with distilled water for 2 min. After dyeing with hematoxylin and eosin in turn as well as mounting with neutral gum, the sections were photographed under an optical microscope (Olympus, Japan) for image acquisition.

### 2.6. TUNEL Staining

The paraffin section specimens for TUNEL staining were taken out and dewaxed with xylene twice (10 min/time) in strict accordance with the instructions of the TUNEL staining kit (Beyotime Biotech). The apoptotic cell count and the total count in 5 nonrepetitive high magnification fields (400×) were randomly selected from each section, and the average percentage of apoptotic cells in each high magnification field was calculated (number of apoptotic cells/total number of cells × 100%).

### 2.7. Oxidative Stress-Related Indicators Assay

The kits used in this experiment were all purchased from Nanjing Jiancheng Bioengineering Institute, China. The freshly preserved rat hippocampus tissues were cut into small tissue pieces with ophthalmic scissors and added with normal saline at the ratio of 1 : 9. The treated hippocampus suspension was then added into 20 mL glass tissue homogenate for grinding up and down and centrifuged at 4°C 3000 × g for 10 min. The obtained supernatant was used as test samples. After incubation with the probe, the relative fluorescence intensity (RFI) was detected by the microplate reader (Bio-Rad, USA). Reactive oxygen species (ROS) activity and malondialdehyde (MDA) content were detected by corresponding detection kits in accordance with the kit instructions.

### 2.8. Inflammatory Factor-Related Indicators Assay

The samples were the same as those used in Section 2.7. The ELISA method was used to determine the absorbance value at 450 nm with a microplate reader. The contents of tumor necrosis factor- (TNF-) *α*, interleukin- (IL-) 6, and IL-1*β* were calculated according to the standard curve. The operating steps followed the kit instructions.

### 2.9. The Contents of Nuclear Factor-*κ*B p65 (NF-*κ*B p65) and Interferon-*γ* (IFN-*γ*) Assay

Nuclear factor kappa-B (NF-*κ*B) is an important transcriptional regulator in cells, usually in the form of P50-P65 isodimer binding to its inhibitor kappa-B (IKB) in an inactive state. NF-*κ*B P65 can release the proinflammatory mediator IFN-*γ*, which participants in chronic inflammatory response and produces physiological changes through complex molecular regulation.

With ophthalmic scissors, the freshly preserved rat hippocampal tissue was cut into small pieces, which were then added with normal saline (tissue : normal saline, 1 : 9). The treated hippocampal tissue suspension was added with 20 mL glass tissue homogenate for grinding up and down and centrifuged (4°C, 3000 × g) for 10 min to obtain the homogenate as the test specimen. NF-*κ*B P65 and IFN-*γ* contents in tissues were detected by ELISA kits (Wuhan Elabscience Biotechnology, China) strictly following the kit instructions.

### 2.10. Western Blot (WB)

The cryopreserved rat hippocampal tissue was cut into fine fragments and weighed and added with 200-400 *μ*L of prepared lysate per 20 mg of tissue mass. The tissue was homogenated with a homogenizer until they were completely decomposed and centrifuged (12000 r/min, 15 min) to collect the supernatant. The BCA method was used to determine the protein content. Thereafter, 50 *μ*g of the protein sample was treated with routine loading, electrophoresis, membrane transfer, and 1 h of sealing with 5% skim milk powder. Then, the closed membrane was moved into the diluted primary antibody working solution for one night of cultivation at 4°C. The primary antibodies included Bcl-2 (1 : 1000, Cell Signaling Technology, USA), Bax (1 : 1000, Cell Signaling Technology, USA), Caspase-3 (1 : 1000, Cell Signaling Technology, USA), JNK (1 : 2000, Cell Signaling Technology, USA), phosphorylated JNK (p-JNK; 1 : 2000, Cell Signaling Technology, USA), p-FoxO3a (1 : 1000, Cell Signaling Technology, USA), and Bim (1 : 1000, Cell Signaling Technology, USA). After eluting with TBST buffer 3 times (5 min/time), it was immersed in horseradish peroxidase-labeled goat anti-rabbit IgG secondary antibody (1 : 3000, Santa Cruz Biotechnology) and incubated in a shaking table at ambient temperature for 2 h, followed by TBST elution 3 times (5 min/time). ECL luminescent solution was dripped on the front of the membrane in a dark room, for detection with an automatic chemiluminescence analyzer. The ImageJ software (version 1.31; National Institutes of Health, USA) was used to analyze the gray value of the band relative to internal reference GAPDH (Cell Signaling, 1 : 1000) for semiquantitative analysis.

### 2.11. Statistical Processing

SPSS20.0 (SPSS Inc., USA) was used for the statistical analysis method. Mean ± standard deviation was used to describe the quantitative data. Two-tailed *t*-test was adopted to analyze the differences between two groups. Differences among multiple groups were analyzed by one-way ANOVA followed by Bonferroni/Dunnett post hoc tests. All the analyses with *P* < 0.05 were considered significant, using *α* = 0.05 as the test standard.

## 3. Results

### 3.1. Behavioral Indicators

All the 24 rats in the Sham group scored 0. The number of rats with a score of 0, 1, 2, 3, and 4 points was 0, 4, 6, 10, and 4, respectively, in the Model group, while it was 0, 8, 9, 4, and 3, respectively, in the L-MT group, 0, 11, 8, 3, and 2, respectively, in the M-MT group, and 0, 11, 9, 3, and 1, respectively, in the H-MT group. The behavioral scores of rats were lower in the L-MT and M-MT groups compared with the Model group (*P* < 0.05), while the behavioral indexes were not significantly different between the H-MT group and Sham group (*P* > 0.05). Twenty rats from the five groups were included, respectively, in the experimental study, as shown in Table 1.

### 3.2. HE Staining

The results of HE staining showed that in the central area of ischemic focus, the neuronal gap and morphology of rats in Sham group were normal, the nuclei were clear, large, and round, and the cytoplasm was light and uniform. The cells in the Model group showed a disappearing normal tissue structure, most of which had reduced size, with loose cytoplasm and pyknotic and deeply stained nuclei, and some presented vacuolar necrosis. The ischemic damage of cells in the L-MT, M-MT, and H-MT groups was notably reduced compared with that in the Model group, with slight edema of cell interstitium, intact cell membrane, and markedly decreased necrotic area. The improvement degree was greater in the M-MT group as compared to the L-MT group, and the improvement degree of M-MT group and H-MT group was similar (Figure 1).

### 3.3. TUNEL Staining

TUNEL staining identified no obvious expression of apoptotic protein in the rat brain tissue in the Sham group. The expression of apoptotic cells increased in the Model group with different volumes and morphology as well as nucleus pyknosis and agglutination, while the apoptotic cells in brain tissue of the L-MT, M-MT, and H-MT groups decreased as compared to the Model group (*P* < 0.05); the H-MT group and the M-MT group had a similar apoptotic cell count (*P* > 0.05) (Figure 2).

### 3.4. Expression of Apoptosis-Related Proteins

Compared with the Sham group, Bcl-2 decreased while Bax and Caspase-3 increased in the Model group (*P* < 0.05); the L-MT, M-MT, and H-MT groups had higher Bcl-2 while lower Bax and Caspase-3 in the rat brain tissue than the Model group (*P* < 0.05). No significant difference was observed in the expression of apoptosis-related proteins between the M-MT and H-MT groups (*P* > 0.05) (Figure 3).

### 3.5. Content of Oxidative Stress-Related Indexes in Rat Brain Tissue

The results showed that compared with the Sham group, the SOD activity in the Model group decreased, while the MDA content and ROS level increased, with statistically significant differences between the two groups (*P* < 0.05). Compared with the Model group, SOD activity in L-MT, M-MT, and H-MT groups increased, while the MDA content and ROS level decreased, and the improvement degree in M-MT group was better than that in the L-MT group, with statistically significant differences (all *P* < 0.05). There was no significant difference between the M-MT group and H-MT group (*P* > 0.05) (Figure 4).

### 3.6. Content of Inflammatory Factors in Rat Brain Tissue

The TNF-*α*, IL-1*β*, and IL-6 levels in the Model group were significantly higher than those in the Sham group (*P* < 0.05). However, in comparison with the Model group, the above inflammatory factors decreased evidently in the L-MT, M-MT, and H-MT groups and were lower in the M-MT group compared with the L-MT group (all *P* < 0.05). No statistical difference was found between the M-MT and H-MT groups (*P* > 0.05) (Figure 5).

### 3.7. Contents of NF-*κ*B P65 and IFN-*γ* in the Rat Brain

ELISA results identified that NF-*κ*B P65 and IFN-*γ* levels in the Model, L-MT, M-HT, and H-MT groups were higher than those in the Sham group (all *P* < 0.05). However, NF-*κ*B P65 and IFN-*γ* in the L-MT, M-MT, and H-MT groups were significantly lower versus the Model group (all *P* < 0.05), and their levels in the M-MT group was lower when compared to the L-MT group (*P* < 0.05) (Figure 6).

### 3.8. Comparison of JNK Expression

WB results revealed no significant difference in the total protein expression of JNK in rat brain tissues among the five groups. The Model group had higher p-JNK contents than the Sham group (*P* < 0.05). p-JNK in the L-MT, M-MT, and H-MT groups decreased significantly versus the Model group. The level of p-JNK was significantly lower in the M-MT group than that in the L-MT group (*P* < 0.05) and was similar in the M-MT and H-MT groups (*P* > 0.05) (Figure 7).

### 3.9. Comparison of FoxO3a and Bim Expression

WB results determined obviously higher p-FoxO3a and Bim in the Model group versus the Sham group (*P* < 0.05). Compared with the Model group, p-FoxO3a and Bim in rat brain tissues in L-MT, M-MT, and H-MT groups decreased, while the M-MT group and H-MT group showed similar FoxO3a and Bim expression (*P* > 0.05). Nevertheless, the levels were lower in the M-MT group when compared to the L-MT group (*P* < 0.05) (Figure 8).

## 4. Discussion

In this study, a rat MCAO model, which has a relatively high success rate with highly similar clinical symptoms, was established by the suture-occluded method [22]. There are many causes of focal cerebral ischemia injury, such as complex cascade injury responses composed of cell apoptosis, free radical damage, oxidative stress, and inflammation [23, 24]. In the state of acute stress, the body's MT concentration decreases, and the function is disorganized. MT has antiapoptosis, anti-inflammation, and antioxidation effects in hypoxic-ischemic brain damage [25]. By observing the pathological changes of brain tissue in rats with focal cerebral ischemia, we found that the nerve cells in the Model group were characterized by the loss of cell structure, hyperchromatism, and cytoplasmic laxity, with vacuolar necrosis in some cells, which indicated the presence of irreversible ischemia and hypoxia injury in the brain tissue during reperfusion injury. However, the brain tissue of rats treated with MT mainly showed swelling of nerve cells, which suggested that the MT can slows down nerve cell necrosis after reperfusion injury to a certain extent. Similar findings have been found by Gou et al. [26], who reported that exogenous MT reduced the pathological damage of brain tissue and suppressed neuronal apoptosis in hypoxic-ischemic rats via the Akt/Nrf2/Gpx4 pathway.

This research also showed that MT can effectively decrease the expression of Bax and Caspase-3, downregulate the levels of NF-*κ*B p65 and IFN-*γ* in brain tissue, and reduce the release of proinflammatory mediators. The activation of inflammatory cells and cascade reaction of inflammatory factors play a dominant role in reperfusion injury [27]. NF-*κ*B p65 contains a processing region that activates transcription and promotes gene transcription and expression in other cells, which is closely related to immune response, inflammatory response, cellular differentiation, proliferation, and apoptosis [28]. NF-*κ*B p65 is shown to activate P38 kinase by releasing the proinflammatory medium IFN-*γ*, which induces cytokine expression and major histocompatibility complexes, inducing apoptosis [29]. The results observed in this study also reflect this mechanism. NF-*κ*B P65 and IFN-*γ* in the Model group, significantly elevated compared with the Sham group, were effectively downregulated by MT. The downregulation level increased with the increase of MT concentration; but the changes that resulted from 40 mg/kg of MT were similar to those caused by medium concentration of MT. Therefore, the optimal MT concentration in this study was 20 mg/kg. In addition, the levels of TNF-*α*, IL-1*β*, and IL-6 in the rat brain tissue in the Model group were significantly higher than those in the Sham group. However, these inflammatory cytokines decreased after intervention with different concentrations of MT, and the decreased levels increased as the concentration increased, which also indicated that MT has an anti-inflammatory effect. Furthermore, we found that MT affected neuronal apoptosis by regulating the JNK/FoxO3a/Bim pathway. As an important stress kinase, JNK can be activated by brain injury in various forms [30]. p-JNK is the activated form of JNK. Phosphorylation of activated JNK stimulates its downstream transcription factors, which triggers Bim of the proapoptotic target gene, thus inducing apoptosis. JNK has been shown to modulate FoxO3a activity in many ways [31], while FoxO3a, a subfamily of the FoxO family discovered in recent years, participates in many pathophysiological processes in vivo, including regulating apoptosis, oxidative stress, and energy metabolism [32]. When focal cerebral ischemia occurs, there will be infiltration of the white blood cells and brain cells (neurons and glia), release of various inflammatory mediators including various cytokines, and production of excessive ROS, resulting in tissue damage [33]. Reducing inflammatory mediators and releasing and controlling oxidative stress through drug action are commonly used to alleviate focal cerebral ischemia. Our results found that after MT intervention, SOD activity increased, MDA content decreased, and ROS level decreased in the Model group. SOD is the main enzyme for removing ROS and other components in the body. When oxidative stress occurs, SOD is constantly consumed, and ROS accumulates in large quantities, resulting in cell damage. Meanwhile, MDA is produced during lipid peroxidation, which reflects the degree of oxidative stress. It can be concluded that MT plays a certain role in antioxidant stress, which may be accomplished through the regulation of oxidative stress produced by the JNK/FoxO3a/Bim signaling pathway. Phosphorylation of FoxO3a can inhibit the activity of FoxO3a and regulate the target gene. Bim, a member of the BH3-only subgroup of the Bcl-2 family, is a vital proapoptotic protein [34]. It has been confirmed that Bim is the downstream gene of FoxO3a, and FoxO3a can bind to Bim promoters to enhance Bim protein expression, thereby initiating the apoptotic process of the mitochondrial pathway [35]. Of note, FoxO3a is identified as a crucial downstream target of MT, mediating the transcriptional regulation of MT-induced proapoptotic Bim [36]. The results of this study also showed that the brain tissue p-JNK, p-FoxO3a, and Bim levels increased significantly in the Model group as compared to the Sham group, while all these indexes in MT-intervened rat brain tissue reduced. Moreover, MT can effectively reduce the expression of Caspase-3 in the rat brain tissue in the Model group. Existing studies have shown that Caspase-3 activation will produce a series of injury reactions, resulting in a large number of delayed apoptosis in infarcts and ischemic penumbra [37]. In the process of ischemic nerve injury, inhibition of Caspase-3 activation can produce neuroprotection, which is also proved by the results of this study.

## 5. Conclusion

To sum up, MT can reduce the release of NF-*κ*B p65 and IFN-*γ* in rats with focal cerebral IRI via the JNK/FoxO3a/Bim pathway, inhibit neuronal apoptosis, and protect the brain against IRI, with anti-inflammatory and antioxidant effects, which has huge implications for clinical prevention and treatment of cerebral IRI. In addition, 20 mg/kg is the optimal melatonin concentration. However, there are still some limitations in this study. Although our finding suggest that the JNK/FoxO3a/Bim pathway might be a key signaling pathways for MT in behavioral and neural regulation, further research is needed on the mode of administration of MT. In addition, this is a preliminary study, and further studies are required to confirm its findings. The prospect of this study was to provide a theoretical basis for the application of MT in clinical work and hope to obtain the clinical significance of MT In focal cerebral IRI.

## Figures and Tables

**Figure 1:** Observation of pathological changes of rat brain tissue by HE staining.

**Figure 2:** Observation of the expression of apoptotic cells in rat brain tissue by TUNEL staining. (a) TUNEL staining of brain tissue of rats in each group. (b) Expression of apoptotic cells in rat brain group in each group. ^∗∗^*P* < 0.01, ^∗∗∗^*P* < 0.001.

**Figure 3:** Expression of apoptosis-related proteins in rat brain tissue. (a) Western blot. (b) Bcl-2 protein expression in brain tissue of rats in each group. (c) Bax protein expression in brain tissue of rats in each group. (d) Caspase-3 protein expression in brain tissue of rats in each group. ^∗∗^*P* < 0.01, ^∗∗∗^*P* < 0.001.

**Figure 4:** Content of oxidative stress related indexes in rat brain tissue. (a) SOD activity. (b) MDA content. (c) ROS level. ^∗^*P* < 0.05, ^∗∗^*P* < 0.01, ^∗∗∗^*P* < 0.001.

**Figure 5:** Content of inflammatory factors in rat brain tissue. (a) Level of TNF-*α*. (b) Level of IL-1*β*. (c) Level of IL-6. ^∗∗^*P* < 0.01, ^∗∗∗^*P* < 0.001.

**Figure 6:** Contents of NF-*κ*B p65 and IFN-*γ* in the brain tissue of rats in each group. (a) NF-*κ*B p65 content. (b) IFN-*γ* content. _∗∗∗_*P* < 0.001.

**Figure 7:** JNK expression in brain tissue of rats in each group. (a) Western blot. (b) JNK expression. (c) p-JNK expression. ^∗∗^*P* < 0.01, ^∗∗∗^*P* < 0.001.

**Figure 8:** Comparison of p-FoxO3a and Bim expression in the brain tissue of rats in each group. (a) Western blot. (b) p-FoxO3a expression. (c) Bim expression. ^∗^*P* < 0.05, ^∗∗^*P* < 0.01, ^∗∗∗^*P* < 0.001.

**Table 1:** Behavioral indicators of rats.

	Behavioral score (*n*)					Behavioral indicators (number of squares climbed)
	0 point	1 point	2 points	3 points	4 points	
Sham (*n* = 24)	24	0	0	0	0	412.3 ± 68.4
Model (*n* = 24)	0	4	6	10	4	329.4 ± 45.1
L-MT (*n* = 24)	0	8	9	4	3	368.7 ± 42.4
M-MT (*n* = 24)	0	11	8	3	2	381.4 ± 51.8
H-MT (*n* = 24)	0	11	9	3	1	385.7 ± 54.2
Sham vs. Model	*P* < 0.0001					*P* < 0.0001
Sham vs. L-MT	*P* < 0.0001					*P* = 0.0127
Sham vs. M-MT	*P* < 0.0001					*P* = 0.0843
Sham vs. H-MT	*P* < 0.0001					*P* = 0.1422
Model vs. L-MT	*P* = 0.1995					*P* = 0.0026
Model vs. M-MT	*P* = 0.0463					*P* = 0.0005
Model vs. H-MT	*P* = 0.0240					*P* = 0.0003
L-MT vs. M-MT	*P* = 0.8314					*P* = 0.3963
L-MT vs. H-MT	*P* = 0.6556					*P* = 0.2606
M-MT vs. H-MT	*P* = 0.9419					*P* = 0.7799

## Data Availability

The labeled dataset used to support the findings of this study is available from the corresponding author upon request.

## References

[1] Knight-Greenfield A., Nario J. J. Q., Gupta A. (2019). Causes of acute stroke: a patterned approach. *Radiologic Clinics of North America*.

[2] Paul S., Candelario-Jalil E. (2021). Emerging neuroprotective strategies for the treatment of ischemic stroke: an overview of clinical and preclinical studies. *Experimental Neurology*.

[3] Herpich F., Rincon F. (2020). Management of acute ischemic stroke. *Critical Care Medicine*.

[4] Stack C. A., Cole J. W. (2018). Ischemic stroke in young adults. *Current Opinion in Cardiology*.

[5] Bhaskar S., Stanwell P., Cordato D., Attia J., Levi C. (2018). Reperfusion therapy in acute ischemic stroke: dawn of a new era?. *BMC Neurology*.

[6] Golts E., Onaitis M. (2021). Commentary: ischemia reperfusion--looking ahead. *The Journal of Thoracic and Cardiovascular Surgery*.

[7] Nakagomi T., Tanaka Y., Nakagomi N., Matsuyama T., Yoshimura S. (2020). How long are reperfusion therapies beneficial for patients after stroke onset? Lessons from lethal ischemia following early reperfusion in a mouse model of stroke. *International Journal of Molecular Sciences*.

[8] Imai T., Matsubara H., Nakamura S., Hara H., Shimazawa M. (2020). The mitochondria-targeted peptide, Bendavia, attenuated ischemia/reperfusion- induced stroke damage. *Neuroscience*.

[9] Naderi Y., Panahi Y., Barreto G. E., Sahebkar A. (2020). Neuroprotective effects of minocycline on focal cerebral ischemia injury: a systematic review. *Neural Regeneration Research*.

[10] Cipolla-Neto J., Amaral F. G. . (2018). Melatonin as a hormone: new physiological and clinical insights. *Endocrine Reviews*.

[11] Wang Y., Jian Y., Zhang X., Ni B., Wang M., Pan C. (2021). *Melatonin Protects Cardiomyocytes from Oxygen Glucose Deprivation and Reperfusion-Induced Injury by Inhibiting rac1/JNK/FoxO3a/BIM Signaling Pathway*.

[12] Zang M., Zhao Y., Gao L. (2020). The circadian nuclear receptor ROR*α* negatively regulates cerebral ischemia- reperfusion injury and mediates the neuroprotective effects of melatonin. *Biochimica et Biophysica Acta (BBA)-Molecular Basis of Disease*.

[13] Irwin M., Tare M., Singh A. (2020). A positive feedback loop of Hippo- and c-Jun-amino-terminal kinase signaling pathways regulates amyloid-beta-mediated neurodegeneration. *Frontiers in Cell and Developmental Biology*.

[14] Vahidinia Z., Azami Tameh A., Nejati M. (2019). The protective effect of bone marrow mesenchymal stem cells in a rat model of ischemic stroke via reducing the c-Jun n-terminal kinase expression. *Pathology-Research and Practice*.

[15] Liu Z., Li C., Wu G. (2020). Involvement of jnk/foxo1 pathway in apoptosis induced by severe hypoxia in porcine granulosa cells. *Theriogenology*.

[16] Bourgeois B., Madl T. (2018). Regulation of cellular senescenceviathe FOXO4-p53 axis. *FEBS Letters*.

[17] Cheng M., Wu X., Wang F., Tan B., Hu J. (2020). Electro-acupuncture inhibits p66shc-mediated oxidative stress to facilitate functional recovery after spinal cord injury. *Journal of Molecular Neuroscience*.

[18] Sun Y.-H., Bu R., Wang Y.-W. (2021). Author correction: validation of efficacy and mechanism of Sanwei-Tanxiang powder in improving myocardial ischemia reperfusion injuries. *Scientific Reports*.

[19] Zhao X., Liu Y., Zhu G. (2019). Sirt1 downregulation mediated manganese-induced neuronal apoptosis through activation of foxo3a-bim/puma axis. *Science of the Total Environment*.

[20] Li D., Li X., Wu J. (2015). Involvement of the jnk/foxo3a/bim pathway in neuronal apoptosis after hypoxic–ischemic brain damage in neonatal rats. *PLoS One*.

[21] Longa E. Z., Weinstein P. R., Carlson S., Cummins R. (1989). Reversible middle cerebral artery occlusion without craniectomy in rats. *Stroke*.

[22] Cao D.-M., Guan Q.-X., Liu Y.-L., Wang S.-M. (2020). Effect of ginsenosides on serous metabonomic profiles in cerebral ischemia-reperfusion rats based on~1h-nmr. *Zhongguo Zhong yao za zhi= Zhongguo zhongyao zazhi=China journal of Chinese materia medica*.

[23] Popa-Wagner A., Petcu E., Capitanescu B., Hermann D., Radu E., Gresita A. (2020). Ageing as a risk factor for cerebral ischemia. Underlying mechanisms and therapy in animal models and in the clinic. *Mechanisms of Ageing and Development*.

[24] Liu H., Wu X., Luo J. (2020). Adiponectin peptide alleviates oxidative stress and nlrp3 inflammasome activation after cerebral ischemia-reperfusion injury by regulating ampk/gsk-3*β*. *Experimental Neurology*.

[25] Cardinali D. P. (2019). An assessment of melatonin’s therapeutic value in the hypoxic-ischemic encephalopathy of the newborn. *Frontiers in Synaptic Neuroscience*.

[26] Gou Z., Su X., Hu X. (2020). Melatonin improves hypoxic-ischemic brain damage through the akt/nrf2/gpx4 signaling pathway. *Brain Research Bulletin*.

[27] Liu H., Wu X., Luo J. (2019). Pterostilbene attenuates astrocytic inflammation and neuronal oxidative injury after ischemia-reperfusion by inhibiting NF-*κ*B phosphorylation. *Frontiers in Immunology*.

[28] Giridharan S., Srinivasan M. (2018). Mechanisms of NF-&kappa;B p65 and strategies for therapeutic manipulation. *Journal of Inflammation Research*.

[29] Wang Q., Zhou X., Zhao Y. (2018). Polyphyllin i ameliorates collagen-induced arthritis by suppressing the inflammation response in macrophages through the nf-*κ*b pathway. *Frontiers in Immunology*.

[30] Bhowmick S., D’Mello V., Abdul-Muneer P. (2019). Synergistic inhibition of erk1/2 and jnk, not p38, phosphorylation ameliorates neuronal damages after traumatic brain injury. *Molecular Neurobiology*.

[31] Kong W., Li C., Qi Q., Shen J., Chang K. (2020). Cardamonin induces G2/M arrest and apoptosis via activation of the JNK–FoxO3a pathway in breast cancer cells. *Cell Biology International*.

[32] Fasano C., Disciglio V., Bertora S., Lepore Signorile M., Simone C. (2019). Foxo3a from the nucleus to the mitochondria: a round trip in cellular stress response. *Cell*.

[33] Zhang T., Li Z., Qin Z. (2021). Neuroprotection of chikusetsu saponin v on transient focal cerebral ischemia/reperfusion and the underlying mechanism. *Phytomedicine*.

[34] Singh P. K., Roukounakis A., Weber A. (2020). Dynein light chain binding determines complex formation and posttranslational stability of the bcl-2 family members BMF and BIM. *Cell Death & Differentiation*.

[35] Liao W., Zhang C., Liu F., Wang W. (2018). Effects of mir-155 on proliferation and apoptosis by regulating FoxO3a/BIM in liver cancer cell line HCCLM3. *European Review for Medical and Pharmacological Sciences*.

[36] Ali T., Rahman S. U., Hao Q. (2020). Melatonin prevents neuroinflammation and relieves depression by attenuating autophagy impairment through foxo3a regulation. *Journal of Pineal Research*.

[37] Wu M., Zhang H., Kai J. (2018). Rapamycin prevents cerebral stroke by modulating apoptosis and autophagy in penumbra in rats. *Annals of Clinical and Translational Neurology*.

